The article "MicroRNA‐155‐3p promotes glioma progression and temozolomide resistance by targeting Six1" was published in 2020. Journal: J Cell Mol Med.

# MicroRNA‐155‐3p promotes glioma progression and temozolomide resistance by targeting Six1

**DOI:** 10.1111/jcmm.15192

**Published:** 2020-03-27

**Authors:** Guangyong Chen, Zhuo Chen, Hang Zhao

**Affiliations:** ^1^ Neurosurgery Department China‐Japan Union Hospital of Jilin University Changchun China

**Keywords:** glioma, miR‐155‐3p, resistance, Six1, temozolomide

## Abstract

The prognosis of glioma is generally poor and is the cause of primary malignancy in the brain. The role of microRNAs has been implicated in tumour inhibition or activation. In several cancers, the Six1 signalling pathway has been found to be aberrant and also relates to the formation of tumours. We analysed the database for expression profiles and clinical specimens of various grades of glioma to assess microRNA‐155‐3p (miR‐155‐3p) expression. The role of miR‐155‐3p in glioblastoma, cell cycle, proliferation, apoptosis and resistance to temozolomide was assessed in vitro through flow cytometry and cell proliferation assays*.* Bioinformatics analyses, and assays using luciferase reporter, and immunoblotting revealed that miR‐155‐3p targets Six1 and that the relationship between glioma and healthy brain tissues was significantly inverse. In rescue experiments, overexpressed Six1 revoked the changes in cell cycle distribution, proliferation and resistance to temozolomide estimated by apoptosis induced by overexpressed miR‐155‐3p. MiR‐155‐3p inhibition reduced glioma cell growth and proliferation in the brain of a mouse model and increased the survival of mice with gliomas. Thus, miR‐155‐3p modulates Six1 expression and facilitates the progression of glioblastoma and resistance to temozolomide and may act as a novel diagnostic biomarker and a target for glioma treatment.

## 1 INTRODUCTION

For past 40 years, glioblastoma multiforme (GBM, or glioma) has shown the highest rate of mortality compared to other brain malignancies and is found to be a commonly occurring primary tumour of the brain.^1^, ^2^ In the United States each year, nearly 20 000 new glioma cases are diagnosed.^3^ Even with available treatments like surgery, radiotherapy and/or chemotherapy, the median survival of glioma patients is only 12 to 14 months for malignant glioma, the most aggressive type.^4^, ^5^ Thus, for ineffective therapy, it is important to explore the process for the growth and advancement of glioma.^6^ An antineoplastic DNA alkylating drug, temozolomide (TMZ), is a chemotherapeutic molecule that freely passes over the blood‐brain barrier and is applied as first‐line therapy to treat glioblastoma with promising results.^7^ It has the capacity to adroitly impede glioma cell proliferation and incite apoptosis.^8^ However, acquired resistance to TMZ is a major barrier in successful treatment.^9^, ^10^, ^11^, ^12^ Therefore, studies aiming to improve the effect of chemotherapy drugs are necessary.

The article "MicroRNA‐155‐3p promotes glioma progression and temozolomide resistance by targeting Six1" was published in 2020. Journal: J Cell Mol Med.

MicroRNAs (miRNAs) are highly conserved, non‐coding, 18‐25 nucleotides long RNA molecules.^13^ They show the capacity to inhibit or activate the advancement of a variety of cancers, such as glioma, and over recent years have exhibited the potential to act as targets for anticancer therapies.^14^, ^15^, ^16^ More than half of the known miRNAs participate in tumorigenesis by targeting tumour suppressor genes or oncogenes directly.^14^, ^17^ Previous studies have shown that miRNAs play a key role in glioma, such as miR‐30a decrease tumorigenicity of glioma stem cells by targeting NT5E‐dependent AKT pathway^18^; miR‐1254 inhibits glioma progression by targeting CSF‐1^19^; and miR‐769‐3p inhibits glioma tumour progression by suppressing ZEB2 and regulating Wnt signalling pathway.^20^ However, the role miR‐155‐3p on gliomas is not well understood.

A member of the Six family, and a homeodomain protein subfamily, transcription factor Six1 (Sine oculis homeobox 1), characteristically possesses a Six‐domain (110‐115 amino acids) and DNA‐binding homeodomain (60 amino acids) and has a vital role in organ development.^21^Mice with Six1‐knockout (KO) die shortly after being born, and embryos of KO are characterized by defective tissues and organs development.^22^ Members of the Six family have the capacity to moderate the specificity of DNA‐binding and activate their target genes at the transcription level by recruiting EYA protein, harbouring phosphatase and transactivation domains.^23^, ^24^

In this study, we showed an increase in the oncogenic capacity of miR‐155‐3p in clinical samples of glioma and correlated with the grades defined by WHO. Further, we found that Six1 is targeted directly by miR‐155‐3p and in an inverse relationship in glioma. We also explored the function of miR‐155‐3p in the regulation of cell cycle, proliferation, apoptosis and resistance to TMZ by targeting Six1 in glioblastoma cells with wild‐type Six1. Our findings implicate miR‐155‐3p as an important biomolecule in the treatment of glioma.

## 2 MATERIALS AND METHODS

### 2.1 Cell lines and TMZ resistance cells generation

The Cell Bank, the Chinese Academy of Sciences (Shanghai, China), provided us with glioma cell lines from humans (LN299, A172, T98, U87 and U251) and healthy human astrocytes. To generate cells resistant to TMZ, U87 and A172 glioma cells were repetitively pulse‐exposed to TMZ. For 6 months, cells were exposed to TMZ at increasing concentrations considering the EC50 values of the cells. From each passage, surviving resistant cell fraction was selected and cultured and was re‐exposed to consecutive TMZ pulse after achieving confluence. The resistant phenotype was sustained by recurrent challenging of TMZ‐resistant cells with 33 μmol/L TMZ. All cell lines were cultured in a 5% CO_2_ atmosphere at 37℃ in Dulbecco's modified Eagle medium (DMEM, Thermo Fisher Scientific) containing 10% foetal bovine serum (FBS, Gibco). TMZ was obtained from Sigma and diluted in DMSO.

The article "MicroRNA‐155‐3p promotes glioma progression and temozolomide resistance by targeting Six1" was published in 2020. Journal: J Cell Mol Med.

### 2.2 Tissue samples from patients

We obtained 20 normal brain tissues and 40 human glioma specimens (II/III and IV) from China‐Japan Union Hospital of Jilin University. The Research Ethics Committee of China‐Japan Union Hospital of Jilin University gave consent to human glioma and healthy brain tissue analyses which were carried out as per guidelines.

### 2.3 Plasmid constructs and stable cell line establishment

Chemical synthesis of miR‐con and miR‐155‐3p mimic was carried out by Ribobio. Plasmid construct harbouring human Six1 was done as per instructions by Genechem. The cDNA of human Six1 was inserted in the pcDNA3 vector, and the recombinant plasmid pcDNA3‐Six1 was generated. Then, seeding was done (2 × 10^5^ cells/well) in 6‐well plates containing complete medium with no antibiotic. After overnight growth, transfection of 100 nmol/L mature miRNA mimics and 7.5 μg plasmids was done for 72 hours into cells along with Lipofectamine 2000 (Invitrogen) as per instructions. The anti‐miR155‐3p or anti‐miR‐con (negative control, anti‐miR) harbouring lentivirus was packaged in 293T cells (human embryonic kidney cells) using the Genechem lentiviral packaging kit for two full days and harvested as per instructions. Transfection of U87 and A172 was done to generate stable cell lines by seeding cells (10 000 cells/well) in 24‐well plates for 24 hours, followed by transfection with lentivirus (0.5 μL; 1 × 10^8^ TU/mL), and then selected on puromycin at 1 μg/mL.

### 2.4 Real‐time PCR

Real‐time PCR was performed as previously research.^25^, ^26^ TRIzol reagent from Life Technologies was used to isolate RNA from fresh tissues and fresh tissues as per the protocol of the manufacturer. Quantitative real‐time PCR was carried out to estimate the level of miR‐155‐3p on the Applied Biosystems ABI StepOne Plus system using the Bulge‐loop™ miRNA qRT‐PCR Primer Kit using appropriate primers (Ribobio). Analyses of data were done by the 2^−ΔΔCt^ process, and the endogenous control was U6. The primers used in this study are listed as follows: miR‐155‐3p, Forward: 5′‐ GACCAACAGCATCACCCTTGA‐3′, Reverse: 5′‐ ACTGCAGGAAGCTATACCAGG‐3′; U6, Forward: 5′‐CTCGCTTCGGCAGCACA‐3′, Reverse: 5′‐AACGCTTCACGAATTTGCGT‐3′.

The article "MicroRNA‐155‐3p promotes glioma progression and temozolomide resistance by targeting Six1" was published in 2020. Journal: J Cell Mol Med.

### 2.5 Western blot assay

Extraction of protein and Western blot assay was done as previously described.^27^, ^28^ In brief, tissues or cells lysed for 0.5 hour on ice in RIPA buffer. Then, the supernatant was collected after centrifuging lysates for 15 minutes at 8000 *g* at 4℃, followed by determination of protein concentrations through bicinchoninic acid assay using the kit from KenGEN (China). Proteins in equal amounts were resolved through SDS‐PAGE (10%) followed by electro‐transfer onto a membrane of polyvinylidene difluoride (PVDF; Thermo Fisher Scientific). Blocking of the membranes was done with 5% non‐fat milk for 60 minutes; then, primary antibodies were added for incubation overnight. Following with secondary antibody incubation for 1 hour, the signal was detected using an ECL detection kit from Thermo Fisher Scientific. The primary antibodies used are listed as follows: cleaved caspase 3 (#9661, Cell Signaling Technology), β‐actin (A5441, Sigma), Six1 (ab211359, Abcam), p21 (ab109520, Abcam), Bcl‐2 (ab32124, Abcam) and bax (ab32503, Abcam).

### 2.6 Assay for cell proliferation

The seeding of cells in their log growth phase (3 × 10^3^ cells/well) was done and maintained in tissue culture plates (96‐well). Assay for cell proliferation was done using the CCK‐8 kit from Sigma at specific time‐points as per instructions. Assay for colony formation was carried out as per a previously published protocol.^29^, ^30^ In brief, cells were plated independently in the wells of tissue culture plates (6‐well). After 2 weeks, colonies that were visible were paraformaldehyde‐fixed (4%) for 20 minutes and stained (crystal violet; 0.1%) for 60 minutes. The efficiency of colony formation was determined as the total colonies with diameter > 0.5 mm. Proliferation assay using EdU (5‐ethynyl‐2'‐deoxyuridine) was done using the kit Molecular Probes EdU‐Alexa imaging from Life Technologies. After two days of transfection, cells were incubated for 60 minutes with EdU (10 μmol/L), followed by fixing, permeabilization and staining with reaction cocktail AlexaFluor 594 and Hoechst 33342 for EdU and cell nuclei, as per provided protocol, and then visualized and the image was acquired under a fluorescent microscope. Each assay was carried out at least thrice.

### 2.7 Analyses of cell cycle

The harvested cells after transfection were given PBS wash and fixed using ethanol (ice‐cold; 70%). These were then resuspended in a from the Cell Cycle Staining Kit from Multi Sciences, China, and incubated in dark for 0.5 hour and then flow cytometrically analysed.

### 2.8 Evaluation of apoptosis

The apoptotic cell number was enumerated using AnnexinV/PI Apoptosis Detection Kit from KeyGEN BioTECH as per the provided instructions. The analysis of apoptotic cells was done on a Gallios Flow cytometer from Beckman, and the results were mentioned as apoptotic cell percentage in comparison with the total cell number.

The article "MicroRNA‐155‐3p promotes glioma progression and temozolomide resistance by targeting Six1" was published in 2020. Journal: J Cell Mol Med.

### 2.9 Luciferase assay

PCR amplification of seed‐matching sites of mutated putative miR‐155‐3p and wild‐type (WT) in Six1 3'‐UTR (untranslated regions) was done using human cDNA and cloned using restriction enzyme *Hind* III and *Sac* I at their sites in the Report vector for pmiRNA from Genechem. Seeding of U87 cells (1 × 10^4^/well) was done in a tissue culture plate (24‐well) and transfected along with 100 ng of WT or mut (mutated) reporter plasmid, 50 nmol/L of miR‐155‐3p mimic or miR‐con as well as 100 ng of Renilla plasmids (internal control). After 24 hours of transfection, the activity of luciferase was evaluated using the Dual‐Luciferase Reporter Assay System from Promega.

### 2.10 Studies on tumour xenografts

All mice‐related experiments were carried out at Model Animal Research Center, China‐Japan Union Hospital of Jilin University as per guidelines of China‐Japan Union Hospital of Jilin University approved for experimental protocols. To carry out xenograft studies, glioma cells (stably expressing 2 × 10^5^ cells) intracranial injection of anti‐miR‐con or anti‐miR‐155‐3p were done in the 4‐ to 6‐week‐old female SCID/NOD mice. The mice harbouring tumours were given oral gavage of TMZ or vehicle (physiologic solution) at week one (three cycles at 100 μmol/L each day for 5 days per week). The measurement of tumours was done every other day. On observing tumour signs, the mice were killed and tumours were extracted at day 19th. These tumours were fixed (10% formalin) and paraffin‐embedded for staining using H&E and immunochemical assessment.

### 2.11 Immunohistochemical analyses

Tumour tissues from nude mouse xenograft were stained for immunohistochemical analyses using antibodies against Six1 as previously reported^31^ and assessed for by analysing cleaved caspase 3. In brief, the sections were deparaffinized using xylene and, subsequently, the ethanol gradient. Citrate buffer at pH 6.0 was used to unmask antigen followed by endogenous peroxidase blocking using hydrogen peroxide (3%). Then, slides were rinsed using phosphate buffer solution (PBS) and kept overnight at 4°C with primary antibodies. Then, slides were processed with ChemMate EnVision Detection Kit (Dako) as per instructions provided.

### 2.12 Statistical analysis

GraphPad Prism 5 software was used for Kaplan‐Meier survival analysis. Each experiment was carried out in triplicate, and standard error of mean or standard deviation and means were analysed for multivariate analysis using ANOVA and compared pairwise using Student's *t* test. For all tests, the significant value considered to be *P* < .05.

The article "MicroRNA‐155‐3p promotes glioma progression and temozolomide resistance by targeting Six1" was published in 2020. Journal: J Cell Mol Med.

## 3 RESULTS

### 3.1 Increase in miR‐155‐3p level in glioma tissues of humans

To analyse the function of miR‐155‐3p in glioma, we analysed the level of miR‐155‐3p in different grades of glioma tissues and found that miR‐155‐3p level was remarkably higher in grade IV (high‐grade) gliomas relative to that in grades II/III (low‐grade gliomas) (Figure 1A). This was also confirmed in the miR‐155‐3p levels in 20 human clinical glioblastoma specimens with higher grade glioma tissues than in 20 low‐grade gliomas and 20 healthy brain tissues (Figure 1B). Clinical glioma and glioma tissues were analysed by the Kaplan‐Meier survival curve using the CGGA database and found that higher expression of miR‐155‐3p (greater than the medium value) correlated with the decline in survival compared to those who contributed samples with low miR‐155‐3p levels, as presented in Figure 1C. We also carried out real‐time PCR to compare miR‐155‐3p levels in the A172, U87, U251, T98 and LN299 glioma cell lines and normal human astrocytes (NHAs) and found high miR‐155‐3p in glioma cells than NHAs (Figure 1D). Our findings indicate that miR‐155‐3p increase in glioma and relative to poor survival.

**Figure 1:** miR‐155‐3p expression is up‐regulated in glioma and correlated with tumour progression. A, CGGA database showing up‐regulated miR‐155‐3p expression in high‐grade glioma tissues compared with that in low‐grade glioma tissues. B, Relative miR‐155‐3p level in glioma tissues was analysed by real‐time PCR. C, Kaplan‑Meier survival analysis from CGGA database showing higher expression of miR‐155‐3p in patients was associated with lower survival rate in glioma. D, The expression of miR‐155‐3p in normal human astrocytes (NHAs) and glioma cell lines was analysed by real‐time PCR. Results were expressed as means ± SD of 3 independent experiments. *P < .05; **P < .01

### 3.2 In vitro analysis shows that miR‐155‐3p activates the growth of glioma cells

To assess the function of miR‐155‐3p in glioma, transient infection of anti‐miR‐155‐3p or anti‐miR‐con was done into A172 and U87 cells expressing high miR‐155‐3p levels and observed significant decline in the miR‐155‐3p level in comparison with anti‐miR‐con‐treated cells (Figure 2A). Furthermore, CCK‐8 assay and colony formation revealed that the decline in miR‐155‐3p expression remarkably inhibited A172 and U87 cell viability relative to the control group (Figure 2B‐E). Similar results were obtained on carrying out cell imaging assay using EDU to assess the miR‐155‐3p effect on proliferation. The anti‐miR‐155‐3p transfected U87 and A172 cells exhibited a lower EDU‐positive rate than the control group (Figure 2F), indicating suppression of glioma cell proliferation on inhibiting miR‐155‐3p. The rate of apoptosis and distribution of cell cycle with miR‐155‐3p knock‐down was also evaluated (Figure 2G). The results of flow cytometry evaluation revealed that miR‐155‐3p knock‐down enhanced the rate of apoptosis, induced cell arrest at the G1/S phase and reduced the percentage of S‐phase cells (Figure 2H,I).

The article "MicroRNA‐155‐3p promotes glioma progression and temozolomide resistance by targeting Six1" was published in 2020. Journal: J Cell Mol Med.

**Figure 2:** miR‐155‐3p promotes glioma growth. A, Relative expression of miR‐155‐3p in A172 and U87 cells was analysed by real‐time RT‐PCR. B, Cell viability assay in A172 cells transfected with anti‐miR‐con or anti‐miR‐155‐3p. C, Cell viability assay in U87 cells transfected with anti‐miR‐con or anti‐miR‐155‐3p. D, Colony formation assay in A172 cells transfected with anti‐miR‐con or anti‐miR‐155‐3p. E, Colony formation assay in U87 cells transfected with anti‐miR‐con or anti‐miR‐155‐3p. F, Edu assay for cells transfected with anti‐miR‐con or anti‐miR‐155‐3p. G, Apoptosis was analysed by flow cytometry in U87 and A172 cells transfected with anti‐miR‐con or anti‐miR‐155‐3p. H, The cell cycle was analysed by flow cytometry in A172 cells transfected with anti‐miR‐con or anti‐miR‐155‐3p. I, The cell cycle was analysed by flow cytometry in U87 cells transfected with anti‐miR‐con or anti‐miR‐155‐3p. Results were expressed as means ± SD of 3 independent experiments. **P < .01

### 3.3 Knock‐down of miR‐155‐3p increases sensitivity of TMZ‐resistant glioma cells

MiR‐155‐3p inhibition as a result of chemotherapy was explored, after transiently transfecting anti‐miR‐155‐3p or anti‐miR‐con into A172/TMZ resistance (TMZ‐R) and U87/TMZ‐resistant cells. The results of real‐time PCR showed a significant reduction in the miR‐155‐3p levels in these cells treated with anti‐miR155‐3p in comparison with cells treated with anti‐miR‐con (Figure 3A). We treated anti‐miR‐155‐3p or anti‐miR‐con stably expressing A172/TR and U87/TR cells with varying TMZ concentrations. A significant increase in chemosensitivity to TMZ was observed after knock‐down of miR‐155‐3p in A172/TR and U87/TR, with a remarkably suppressed cell viability, exhibiting an inverse relationship with TMZ concentrations relative to the observations in miR‐con group (Figure 3B,C). Similar results were observed on cell proliferation by evaluating the effect of miR‐155‐3p along with TMZ by EDU cell image and colony formation assays (Figure 3D‐F). Our findings also shown that miR‐155‐3p inhibitor enhances TMZ‐induced apoptosis in the TMZ resistance cells (Figure 3G, H). Further, an increase in cleaved caspase 3 in association with the rate of apoptosis was observed through Western blotting (Figure 1I).

The article "MicroRNA‐155‐3p promotes glioma progression and temozolomide resistance by targeting Six1" was published in 2020. Journal: J Cell Mol Med.

**Figure 3:** miR‐155‐3p knock‐down sensitizes resistant glioma cells to TMZ. A, Relative miR‐155‐3p level was analysed by real‐time PCR in A172/TR and U87/TR cells. B, Cell viability assay in A172/TR cells transfected with anti‐miR‐con or anti‐miR‐155‐3p and treated with increasing dose of TMZ. C, Cell viability assay in U87/TR cells transfected with anti‐miR‐con or anti‐miR‐155‐3p and treated with increasing dose of TMZ. D, Edu assay of U87/TR and A172/TR cells transfected with anti‐miR‐con or anti‐miR‐155‐3p and treated with 100 μmol/L TMZ for 48 h. E, Colony formation assay in A172/TR cells transfected with anti‐miR‐con or anti‐miR‐155‐3p and treated with increasing dose of TMZ. F, Colony formation assay in U87/TR cells transfected with anti‐miR‐con or anti‐miR‐155‐3p and treated with increasing dose of TMZ. G, Apoptosis was analysed by flow cytometry in A172/TR cells transfected with anti‐miR‐con or anti‐miR‐155‐3p and treated with 100 μmol/L TMZ after 48 h. H, Apoptosis was analysed by flow cytometry in U87/TR cells transfected with anti‐miR‐con or anti‐miR‐155‐3p and treated with 100 μmol/L TMZ after 48 h. I, Western blotting of indicated proteins in U87/TR cells transfected with anti‐miR‐con or anti‐miR‐155‐3p and treated with 100 μmol/L TMZ after 48 h. Results were expressed as means ± SD of 3 independent experiments. **P < .01

### 3.4 miR‐155‐3p directly targets Six1 in glioma cells

The bioinformatics analytical tool TargetScan was employed to comprehend the activity of miR‐155‐3p and its potential target genes in glioblastoma and found matching the 3′‐UTR of Six1 matched and the miR‐155‐3p sequence, as confirmed by transfecting the luciferase report vector construct harbouring the Six1 3′‐UTR in U87 cells (Figure 4A). Nearly 80% reduction in relative luciferase activity of WT‐Six1 by miR‐155‐3p mimics was observed, whereas minimal inhibition was observed in cells transfected Mut‐Six1 luciferase reported (Figure 4B,C) implicating that Six1 is targeted directly by miR‐155‐3p. We further observed that miR‐155‐3p knock‐down in both A172 and U87 glioma cells increased endogenous Six1 levels and its downstream proteins, but no notable change was observed in the transcript levels (Figure 4D), thus indicating the inhibition of Six1 by miR‐155‐3p at the translational and not transcription level. Then, A172 cells were cotransfected with miR‐con or miR‐155‐3p, in the absence or presence of Six1 plasmid for more clarity on the synergistic effects of Six1 (Figure 4E). Our findings also showed low level of Six1 in glioma cells than NHAs (Figure 4F). In addition, Six1 levels were measured in 20 high‐grade and 20 low‐grade tissues of glioma and 20 non‐cancerous tissues of the brain, and significant decline in Six1 proteins levels in low‐grade or high‐grade glioma specimens was observed compared with that in normal brain tissue (Figure 4G). Next, Pearson's correlation analysis between Six1 protein and miR‐155‐3p levels in tissues revealed an inverse relationship between Six1 levels and miR‐155‐3p expression (Figure 4H).

The article "MicroRNA‐155‐3p promotes glioma progression and temozolomide resistance by targeting Six1" was published in 2020. Journal: J Cell Mol Med.

**Figure 4:** miR‐155‐3p targeting Six1 in glioma. A, The predicted base pairing in miR‐155‐3p and Six1 from TargetScan. B, Validation of targeting relation between miR‐155‐3p and Six1 through dual‐luciferase reporter assay in A172 cells. C, Validation of targeting relation between miR‐155‐3p and Six1 through dual‐luciferase reporter assay in U87 cells. D, Western blotting of Six1 in A172 and U87 cells transfected with indicated miR‐155‐3p or anti‐miR‐155‐3p. E, Western blotting of Six1 in A172 cells transfected with miR‐155‐3p with or without Six1 overexpression plasmid. F, The mRNA level of Six1 was higher in glioma cell lines than that in normal cell line NHAs. G, Relative mRNA level of Six1 in glioma tissues was analysed by real‐time PCR. H, Spearman correlation analysis of Six1 and miR‐155‐3p level in glioma tissues. Results were expressed as means ± SD of 3 independent experiments. **P < .01

### 3.5 The oncogenic effect of miR‐155‐3p was abrogated by reintroducing Six1

After transfecting A172 and U87 cells with miR‐155‐3p (Figure 5A), the role of Six1 was evaluated on the growth‐promoting role of miR‐155‐3p in glioma cells by cotransfecting miR‐155‐3p mimics and human Six1 plasmids into A172 and U87cells. As shown in Figure 5B‐H, the activities of miR‐155‐3p on cell cycle distribution and cell proliferation were inhibited by overexpressing Six1. Moreover, increased Six1 expression in A172 and U87 cells remarkably impeded proliferation and facilitated arrest at G1/S cell cycle. A reduction in BAX and p21 expression was rescued by abnormal Six1 expression and rescued miR‐155‐3p mimic‐induced enhanced BAX and p21 levels in both A172 and U87 cells (Figure 5I‐J). Thus, the function of Six1 is targeted by miR‐155‐3p in glioma cells.

**Figure 5:** Six1 reintroduction reverses the promotional effect of miR‐155‐3p. A, Relative expression of miR‐155‐3p in A172 and U87 cells was analysed by real‐time PCR. B, Cell viability was analysed in A172 cells transfected with miR‐con or miR‐155‐3p with or without Six1 overexpression. C, Cell viability was analysed in U87 cells transfected with miR‐con or miR‐155‐3p with or without Six1 overexpression. D, Edu assay in A172 cells transfected with miR‐con or miR‐155‐3p with or without Six1 overexpression. E, Colony formation was analysed in A172 cells transfected with miR‐con or miR‐155‐3p with or without Six1 overexpression. F, Colony formation was analysed in U87 cells transfected with miR‐con or miR‐155‐3p with or without Six1 overexpression. G, Cell cycle was analysed by flow cytometry in A172 cells transfected with miR‐con or miR‐155‐3p with or without Six1 overexpression. H, Cell cycle was analysed by flow cytometry in U87 cells transfected with miR‐con or miR‐155‐3p with or without Six1 overexpression. I, Western blotting of indicated protein in A172 cells transfected with miR‐con or miR‐155‐3p with or without Six1 overexpression. J, Western blotting of indicated protein in U87 cells transfected with miR‐con or miR‐155‐3p with or without Six1 overexpression. Results were expressed as means ± SD of 3 independent experiments. *P < .05; **P < .01

The article "MicroRNA‐155‐3p promotes glioma progression and temozolomide resistance by targeting Six1" was published in 2020. Journal: J Cell Mol Med.

### 3.6 Six1 reintroduction rescues miR‐155‐3p‐mediated TMZ resistant

The role of Six1 on miR‐155‐3p‐mediated TMZ resistance in glioma cells was assessed by cotransfecting human Six1 plasmids and mimics of miR‐155‐3p into A172 and U87 cells. MiR‐155‐3p‐mediated stimulation of proliferative capacity and apoptotic inhibition was repressed by overexpressing Six1 in the medium containing TMZ. Further, increased Six1 alone significantly facilitated apoptosis and suppressed proliferation in A172 and U87 cells in medium containing TMZ (Figure 6A‐D), in addition to a decline in cleaved caspase 3 protein (Figure 6E‐F). Thus, Six1 overexpression reverses resistance to TMZ in glioma cells with high levels of miR‐155‐3p.

**Figure 6:** Six1 reintroduction rescues the TMZ‐resistant effect of miR‐155‐3p. A, Cell viability of A172 cells transfected with miR‐con or miR‐155‐3p with or without Six1 overexpression was treated with increasing dose of TMZ. B, Cell viability of U87 cells transfected with miR‐con or miR‐155‐3p with or without Six1 overexpression was treated with increasing dose of TMZ. C, Colony formation assay of A172 cells transfected with miR‐con or miR‐155‐3p with or without Six1 overexpression was treated with increasing dose of TMZ. D, Colony formation assay of U87 cells transfected with miR‐con or miR‐155‐3p with or without Six1 overexpression was treated with increasing dose of TMZ. E, Western blotting of cleaved caspase 3 of A172 cells transfected with miR‐con or miR‐155‐3p with or without the Six1 overexpression treated with 100 μmol/L TMZ for 48 h. F, Western blotting of cleaved caspase 3 of U87 cells transfected with miR‐con or miR‐155‐3p with or without the Six1 overexpression treated with 100 μmol/L TMZ for 48 h. Results were expressed as means ± SD of 3 independent experiments. **P < .01

The article "MicroRNA‐155‐3p promotes glioma progression and temozolomide resistance by targeting Six1" was published in 2020. Journal: J Cell Mol Med.

### 3.7 Knock‐down of miR‐155‐3p inhibits the growth of tumours and increases TMZ sensitivity

Further, in an in vivo experiment on the U87 xenograft mice model (6 mice/group), the introduction of xenografted tumours was done by U87 glioma cells either with anti‐miR‐con or with anti‐miR‐155‐3p, in the presence or absence of TMZ. The anti‐miR‐155‐3p group exhibited a significant intracranial tumour volume reduction in comparison with the anti‐miR‐con group in these models (Figure 7A,B). Anti‐miR‐155‐3p sensitized U87 tumour to TMZ (Figure 7A,B). At the study end, Western blotting and cleaved caspase 3 staining revealed a remarkable increased caspase 3 activation in the combination group (Figure 7C,F). Consistent with in vitro results, Western blotting and immunohistochemistry revealed enhanced expression of Six1 in anti‐miR‐155‐3p tumours (Figure 7D,E). Thus, miR‐155‐3p activates the growth of glioma cells and increases the sensitivity of tumours to TMZ in vivo.

**Figure 7:** miR‐155‐3p inhibition sensitizes TMZ in vivo. A, U87 cells pre‐treated with a lentivirus expressing anti‐miR‐155‐3p or anti‐miR‐con were injected in both flank of nude mice. Tumour volume was calculated every two days. B, Tumour weight was analysed at end of the experiment. C, Western blotting of cleaved caspase 3 in indicated tumours. D, Western blotting of Six1 in indicated tumours. E, Representative immunohistochemical images of Ki‐67 in anti‐miR‐155‐3p and the anti‐miR‐con transfected tumours. Scale bar: 25μm. F, IF staining of cleaved caspase 3 in indicated tumours. Scale bar: 25μm

## 4 DISCUSSION

MicroRNAs have been indicated in activating or inhibiting a range of activities associated with oncogenes, such as cell cycle and apoptosis, proliferation and resistance to TMZ.^32^, ^33^ Abnormal regulation of miRNA expression has been detected in several tumours, including that of the brain such as glioma and its subtype, the aggressive glioblastoma.^34^ MiRNAs also play a key part in advanced stages of cancer as tumour suppressors or activators.^35^ Significantly elevated miR‐155 was detected in tissues of breast cancer, and its high levels statistically indicated an association with the positive status of lymph node metastasis, especially for breast cancer patients with the triple‐negative result.^36^ Correspondingly, detected significantly higher miR‐155 expression in tumour tissues than that in the matched non‐tumour tissues, with a close relation to advanced clinical TNM stage, lymph node positivity and higher index of proliferation.^37^ Further, miR‐155 knock‐down clearly reduced viability and promoted apoptosis of breast cancer cells.^38^, ^39^ Likewise, in this study, we found increased miR‐155‐3p in a higher grade glioblastoma and its knock‐down in glioblastoma cells stalled proliferation, induced apoptosis, led to arrest of the cell cycle and resistance to TMZ. A decline in miR‐155‐3p level in nude mice tumour xenografts reduced the speed of tumour growth and increased the survival time of these mice. We could also show that miR‐155‐3p overexpression in glioma cells caused decrease in Bax and p21 and expression by directly targeting the Six1 3′‐UTR.

The article "MicroRNA‐155‐3p promotes glioma progression and temozolomide resistance by targeting Six1" was published in 2020. Journal: J Cell Mol Med.

Six1 regulates the development of several organs by inhibiting apoptosis and modulating cell cycle regulators.^40^ Mouse embryos with Six1^−/−^ exhibit defects in the survival of the precursor cells of multiple organs as well as in proliferation and, ultimately, die during birth.^22^ As an oncogene, Six1 is overexpressed in colorectal cancer, breast cancer, pancreatic cancer and squamous cell carcinoma of the oesophagus and is associated with the growth, advancement and prognosis of multiple tumours.^21^, ^41^, ^42^, ^43^ Concurrently, here, we confirmed the up‐regulation of Six1 at both transcript and protein levels in patients when compared with healthy individuals. The cell lines also exhibited high levels of Six1. Previous studies demonstrated that Six1 promoted cell proliferation, migration and invasion in endometrial cancer.^44^, ^45^ In addition, it has been reported that Six1 up‐regulation induces cancer cell EMT. Six1 up‐regulation leads to EMT via the activation of zinc‐finger E‐box binding homeobox 1.^46^ Particularly, a recent study demonstrated that Six1 is overexpressed in endometrial carcinoma and promotes the malignant behaviour of cancer cells via ERK and AKT signalling.^47^ We demonstrated in this study that Six1 could be developed as a therapeutic target for glioma patients because of its vital roles in glioma.

Our results show therefore the tumour‐promoting activity of miR‐155‐3p through various mechanisms, including apoptotic inhibition, tumour cell growth promotion and initiation of cell cycle arrest. While the Six1 level decreased in U87 and A172 cells with miR‐155‐3p transfection. While U87 and A172 cells are Six1 mutation cell lines and cell lines U87 and A172 were of Six1 wild‐type, MiR‐155‐3p decreased expression of Six1 in U87 and A172 cells could not efficiently promote U87 and A172 cells growth. Here, miR‐155‐3p knock‐down enhanced TMZ sensitivity in human glioma cells and induced apoptosis in glioma cells. Nevertheless, Six1 is not the only mode of affecting TMZ resistance in glioma, and some potential ways independent of Six1 mutation have possibly not been discovered. These outcomes will guide us to study TMZ resistance in glioma. Thus, we hypothesize that the anti‐miR‐155‐3p and TMZ combination could be a promising treatment strategy to suppress glioma growth.

The article "MicroRNA‐155‐3p promotes glioma progression and temozolomide resistance by targeting Six1" was published in 2020. Journal: J Cell Mol Med.

In conclusion, our current study provides significant insights into tumorigenesis and miR‐155‐3p relationship in human glioma. We could show that miR‐155‐3p acts as a promoter of tumours by targeting Six1 and inhibiting Six1‐associated pathways. Interestingly, we found that the glioma cell resistance to TMZ treatment is enhanced by miR‐155‐3p treatment. Despite being in preliminary stages of development, miRNA‐based therapeutics are promising, and our findings give a potential indication of the role of miR‐155‐3p as potential prognostic/diagnostic marker and a possible target for glioma treatment.

## CONFLICT OF INTEREST

The authors declare that they have no conflict of interest.

## AUTHOR CONTRIBUTION

GC, ZC and HZ designed the study. GC and HZ collated the data and carried out data analysis. HZ generated the draft of the manuscript. All authors have read and approved the final submitted manuscript.

## Data Availability

The data that support the findings of this study are available from the corresponding author upon reasonable request.
